# Agricultural Economic Evidence and Policy Prospects under Agricultural Trade Shocks and Carbon Dioxide Emissions

**DOI:** 10.1155/2022/5988270

**Published:** 2022-08-24

**Authors:** Jian Kang, Minjuan Zhao

**Affiliations:** ^1^College of Economics and Management, Northwest A & F University, Yangling, Shaanxi 712100, China; ^2^Shaannan Eco-Economy Research Center, Ankang University, Ankang, Shaanxi 725000, China

## Abstract

With the development of the market economy, agricultural trade has become more and more significant for the development of the agricultural economy, which has triggered people's further thinking and exploration on the impact of agricultural trade on agricultural carbon emissions. This paper takes the measurement of trade implied carbon as the carbon dioxide emission index under the impact of agricultural trade and analyzes the impact of trade implied carbon and implied carbon balance on carbon emission. Taking the impact of Sino-US agricultural trade as an empirical background, this paper measures the impact of environmental changes in agricultural trade opening on China's agricultural development and its carbon emissions, so as to predict changes in China's regional agricultural carbon emissions performance. After calculation, it is found that the scale of China's exports has decreased by 0.089%, which is lower than the decline of 0.361% in the United States. The trade conflict has a significant impact on China's import and export structure. Under the scenario of mutual tariffs on agricultural products, China's exports to the United States are expected to decrease by 6.28%, while China's imports from the United States decreased by 13.02%. The Sino-US agricultural trade dispute will reduce China's carbon emissions by 0.013% and the United States' carbon emissions by 0.024%, which is related to the negative impact on the economy. Improving the performance of agricultural carbon emissions is not only the need for the green and sustainable development of the agricultural economy but also conducive to improving the international competitiveness of agricultural products.

## 1. Introduction

China's economic construction is gradually in line with the world, and the economic status has been continuously improved. Behind the great achievements, it is also necessary for people to become more rational and sober. The development imbalance between regions or between urban and rural areas is becoming more serious. The quality and structural level of development are low. The existing agricultural production efficiency is still low, and the driving force and level of rural economic development need to be improved. The income gap between rural residents and urban residents has further widened and most of them are still in poverty. Therefore, the key to developing the rural economy, promoting agricultural development, and improving farmers' income is to scientifically and effectively handle the problems of rural areas, agriculture, and farmers. The development of low-carbon agriculture in China has potential, motivation, and pressure. Therefore, in order to fulfill the responsibility of a big country, it is necessary to develop a low-carbon economy. To develop a low-carbon economy, people must give priority to the development of modern low-carbon agriculture. Therefore, it is of great significance to study the low-carbon development of agricultural trade.

There is a balanced relationship between agricultural economic development and social and ecological environment. Li et al. identified and quantified agricultural residues [1]. Cole and Xiong studied agricultural insurance (AI) schemes in developing countries [2]. Mason et al. believed that the fertilizer subsidy program will become a policy [3]. Luo et al. compared the decoupling of China's agricultural carbon dioxide emissions and agricultural output in different regions and years [4]. Li et al. believed that crop prices are the most sensitive influencing factors [5]. Their study of agricultural economics did not take environmental factors into account. This article will locate how agricultural trade conflicts play out in the agricultural economy, with a view to discovering its value in this area.

The agricultural trade shock has an important impact on the fluctuation of the agricultural economic cycle. Eor analyzed the agricultural production factors of various countries [6]. Udoh and Adelaja used regression analysis to evaluate agricultural trade data [7]. Li and Andreosso-O'Callaghan analyzed and compared the advantages of EU27 countries (excluding the UK) and China [8]. Mizik et al. aimed to analyze the comparative advantage model of the commonwealth of independent states agriculture [9]. Widyasari et al. forecast future direction and trends in agricultural trade [10]. To a certain extent, agricultural economic growth can reduce the growth rate of carbon dioxide emissions. This paper will make further research on the impact of agricultural trade.

At present, there are three main means to reduce embodied carbon emission: management emission reduction, technical emission reduction, and structural emission reduction. This paper will study in detail the impact of country sources, product distribution, and transportation means of embodied carbon emissions in international trade in agricultural products. It will provide constructive decision-making suggestions for optimizing the structure of agricultural trade, further improving the production of agricultural products and the low-carbon development of the industrial structure. The research method of this paper is mainly based on the multi-regional input-output model (MRIO), which can make up for the current agricultural carbon footprint research that only focuses on the carbon emissions in production or logistics transportation, while ignoring the impact of agricultural import and export trade on carbon footprint. In this way, a more comprehensive method is constructed to measure the scale, country and product distribution of China's agricultural trade embodied carbon in the context of agricultural trade globalization. It is found that the embodied carbon of China's agricultural export trade increased by 118.69%, and the trade volume increased from 4.609 billion yuan to 16.275 billion yuan during the same period, with an increase of 253.10%.

## 2. Agricultural Economics Analysis

### 2.1. Agricultural Economic Policy

With the continuous improvement of China's agricultural policy, China's economy has maintained a rapid and steady growth. Through the analysis of the influencing factors such as the total power of agricultural machinery, the amount of fertilizer application, and labor input, the government can better guide the government to clarify the purpose of the special agricultural subsidy funds, such as subsidies for agricultural machinery and motivation. Positive policies that benefit farmers can promote the development of agriculture, further guide farmers' motivation for farming, and are also beneficial to agricultural income and improve the overall quality of life of farmers. This can also enhance the pertinence of the government's agricultural expenditure and the efficiency of the use of funds [11, 12]. Agricultural production activities directly affect the natural environment. With the development of chemical agriculture and mechanical agriculture, agriculture has become an important source of greenhouse gas emissions.

## 3. Agricultural Trade and Low-Carbon Economy

The main features of a low-carbon economy are “low consumption, low emissions, and low pollution”. In the partial equilibrium model of green agricultural trade policy, if a country's trade of a certain green agricultural product is so large that it affects the world market price, it is called a major trading country of this agricultural product. In reality, it is often a developed country and tends to adopt positive support policies. Correspondingly, countries that cannot cause significant fluctuations in world market prices are called small trading countries of such agricultural products, which are often in developing countries that tend to adopt negative support policies. The large country model is used for the positive support policy of agricultural trade, and the small country model is used for the negative support policy of agricultural trade. Through the analysis of the green agricultural trade support policies of developing and developed countries, the government's intervention policies may appear to be too costly in terms of national economic welfare. This exacerbates price fluctuations in the world market, distorts the flow of agricultural trade, and leads to an imbalance in the allocation of world resources [13]. China is not only relatively scarce in land resources, but also has a high cost of land use. It should reduce the production scale of land-intensive agricultural products and increase their imports, so as to improve the efficiency of resource allocation.

Agricultural production emits large amounts of greenhouse gases such as carbon dioxide, methane, and nitrous oxide. Among them, carbon dioxide mainly comes from the use of energy. Methane mainly comes from ruminant animal feeding, rice cultivation, and animal excretion. Nitrous oxide mainly comes from the use of chemical fertilizers and animal manure. The particularity of agriculture is determined by its own characteristics. That is, agricultural production activities will not only emit a large amount of greenhouse gases to cause climate change, but more importantly will be adversely affected by climate change to a greater extent. The essence of low-carbon agriculture is the scientific and rational use of chemical fertilizers and energy, optimization of planting technology and structure, etc., in order to achieve the “three lows” development of agriculture, so that the environment and agricultural economic development achieve harmony and unity. Low-carbon agriculture is the embodiment of a low-carbon economy in the process of agricultural development, which is an indispensable part of the process of low-carbon economic development. The impact of agricultural trade liberalization on the agricultural environment is shown in Figure 1 [14].

## 4. Calculation Model of Carbon Embodied in Trade

With the increasing scale of foreign trade in agricultural products, the greenhouse gas emissions caused by foreign trade cannot be underestimated for the reduction of greenhouse gas emissions from agricultural production. Compared with a single factor, this paper not only examines CO_2_ output from the perspective of agriculture, but also examines the impact of different input factors and their alternative factors on carbon emission efficiency. Therefore, the measurement of agricultural CO_2_ needs to be more comprehensive. Based on the total factor productivity theory, this paper takes the expected output of agricultural carbon emissions as the expected performance of carbon measurement. Some scholars take other pollutants as unexpected outputs to measure and measure carbon emissions. This paper will measure the performance of agricultural carbon emissions from the perspective of agricultural total factor productivity.

Without considering international trade, the total output of a sector in a country can satisfy all intermediate and final demands for the products produced by that sector. Therefore, the basic model of input-output analysis can be defined as follows [15]:

(1) $$\begin{array}{c} \sum_{j}^{m}a_{ij}x_{j}+y_{j}=x_{i}. \end{array}$$

In formula (1), *a*_*ij*_ represents the direct emission factor. The model can detect the magnitude of the variable response value after a given system shock, the direction of change (positive and negative), and the number of cycles affected by the system after the shock.

The carbon dioxide emission coefficient of each energy source per unit mass is given as follows:

(2) $$\begin{array}{c} AC_{i}=C_{i}*\left(1+H_{i}\right). \end{array}$$

In formula (2), AC is the adjusted CO_2_ emission factor [16].

The theoretical analysis model of the relationship between agricultural carbon emissions and agricultural economic growth is shown in Figure 2. Through the analysis of green agricultural trade support policies in developing and developed countries, the government's intervention policies may appear too costly in terms of national economic welfare. This exacerbates price fluctuations in the world market, distorts the flow of agricultural trade, and leads to an imbalance in the allocation of world resources. In economically developed countries, people's institutional demands on the environment are stronger, and they begin to put pressure on the government. They force the government to adopt the trade policy supply that serves the environmental goal, leading to the change of the environmental protection system and the trade support system, which becomes a typical induced system change. In the process of sustainable agricultural development, it is currently facing three pressures: the lack of resources, ecological pollution, and the international commitment to reduce carbon emissions.

## 5. Data Source and Processing

The empirical analysis of the MRIO model (It is a regional input-output model which is an input-output model prepared for a region and a component of the overall input-output model.) requires three parts of data, namely, the import and export trade volume between China and its trading partners, the direct carbon emission coefficient by industry, and the input-output table. The import and export trade volume data between China and its trading partners is taken from the 0ECDSTAN Bilateral Trade Database (BTD), and the industry is classified with reference to the International Trade Classification Standard (ISICRev4.0). The carbon direct emission coefficient and input-output table data by industry are taken from the WIOD database. This paper adopts the estimation method based on fuel classification. In specific operations, the total amount of carbon dioxide emissions is obtained by summing up the estimated carbon dioxide emissions from various types of energy consumption, and its calculation formula is given as follows [17]:

(3) $$\begin{array}{c} C=\sum \left(AC_{i}*EC\right). \end{array}$$

In formula (3), *C* is the total carbon dioxide emissions, and *EC* is the total energy consumption.

## 6. Evaluation of the Transformation of Agricultural Economic Growth Mode

The large-scale management of farmland not only is reflected in the increase of input of production factors and the progress of technical level, but also makes the allocation ratio of various production factors better. The combination of various factors has the highest production efficiency under a certain technical level. That is to say, agricultural large-scale production reduces marginal production costs, increases scale returns, and improves agricultural production efficiency by expanding crop planting area and rationally matching capital, technology, and human capital investment. This paper uses the total factor productivity method to evaluate the agricultural economic growth mode. The main input elements of agricultural economic growth include capital, labor, and land, so its growth rate equation is given as follows [18]:

(4) $$\begin{array}{c} G=G_{A}+\delta G_{M}+\mu G_{N}+\varepsilon G_{P}. \end{array}$$

In formula (4), *G* represents the growth rate of agricultural output, and GA represents the total factor growth rate.

This paper adopts the total agricultural output value as an indicator reflecting the total agricultural output. In the process of traditional agricultural growth, the expansion of land use has always been the most important factor in agricultural growth. With the advancement of technology, the improvement of the level of agricultural material and technical equipment, the increasing population and the contradiction between the non-renewable land resources have become prominent. The growth of modern agriculture mainly depends on the improvement of the depth of land use.

## 7. Evaluation of the Process of Transformation of Agricultural Economic Growth Mode

Quantitative evaluation of the transformation of agricultural economic growth mode must be based on the actual situation and the method chosen. The deviation value is equal to the difference between the actual value and the target value, and its main meaning is the gap between the indicators of agricultural growth mode and the daily target of primary intensive management. The dispersion method comprehensively reflects the degree to which the evaluation index of the agricultural economic growth mode approaches the standard value, that is, the comprehensive level of the achieved degree that the agricultural growth mode has changed from extensive to intensive. The dispersion method can test whether the difference between the means of two or more samples is statistically significant. The formula for calculating the dispersion level of each indicator is given in as follows [19]:

(5) $$\begin{array}{c} G=\sum_{i=1}^{3}\left(\sum_{j=1}^{n}X_{ij}*w_{ij}\right). \end{array}$$

In formula (5), *G* is the agricultural growth intensification level index.

With the acceleration of urbanization in China in recent years, urbanization has promoted the adjustment of agricultural economic structure. First, urbanization integrates the current rural production factors and resources. On the one hand, many farmers migrated to cities and towns, making land resources more concentrated. Many of the original small-scale farmers with decentralized operations have been transformed into large-scale farmers and new production forms such as farms and cooperatives. The adjustment of the agricultural structure requires a certain amount of land as support, so urbanization meets the requirements of agricultural structure adjustment for land. Second, in the past, the agricultural products produced by farmers under the family based production method were often small in scale and complete in variety, but the emergence of urbanization made farmers produce specific agricultural products in a targeted manner. There is demand among farmers who produce different agricultural products, which promotes the specialized production and regionalization of agriculture. This change makes the production factors recombine and gives play to the regional comparative advantage, promoting the optimization and adjustment of the agricultural structure. In this paper, the ADF unit root test method is used to test the two variables, LnAI and LnTAP, to judge their single integer order. In the ADF test, if the series is stationary, there is no unit root. Otherwise there is a unit root. The method of ADF unit root test is given as follows [20]:

(6) $$\begin{array}{c} W_{t}=\alpha t+\beta +\delta W_{t-1}+\theta_{t-i}+\varepsilon_{i}. \end{array}$$

In formula (6), *α*, *β*, *δ*, and *θ* are parameters; *t* is a time trend factor; *ε* is a random error term.

## 8. Results of Agricultural Economy

Among the proportions of various agricultural products in 2019, vegetable exports accounted for 20.5%. Aquatic products exports accounted for 30%. Fruit exports accounted for 10.4%. Livestock products exports accounted for 9.4%. Beverage exports accounted for 6.3% (The statistics of vegetables, aquatic products, fruits, livestock products, and beverages are shown in Figure 3(a)). Exports of food products accounted for 2.5%. Oilseed exports accounted for 2.3%. Sugar exports accounted for 2.3%. Nut exports accounted for 1.6%. The total export of other agricultural products accounted for 18.6%. The total exports of fruits and vegetables accounted for 30.9% (Grain products, oilseeds, sugar, nuts, and other agricultural products are shown in Figure 3(b)). China's labor resources are abundant but land resources are scarce. According to the theory of comparative advantage, with the continuous improvement of agricultural trade openness, the agricultural production structure will also change. Agricultural infrastructure inputs affect trade, transportation costs, etc. The level of agricultural infrastructure has a certain impact on the scale of trade, and then the trade will have different effects on agricultural carbon emissions performance due to the different levels of infrastructure in each region. The low-carbon agriculture theory is the demand of this research and the support of this paper. The total factor productivity theory is the theoretical basis for the calculation and decomposition of carbon emission performance.

The import proportion of China's agricultural products is aquatic products (9%), vegetable oil (5.7%), beverages (5.2%), grain (5.2%), fruit (5%) (The statistics of imported aquatic products, vegetable oils, beverages, grains, and fruits are shown in Figure 4(a)), cotton and linen silk (2.4%), grain products (1.6%) (%), and other products (11.4%). Oilseeds and livestock products together account for more than 50% of imported agricultural products. The source countries of China's imports are mainly concentrated in some European and American countries (The statistics of imported cotton and linen silk, grain products, other products, oilseeds, and livestock products are shown in Figure 4(b)).

The content of sustainable agriculture theory includes: respecting nature, protecting agricultural resources and environment, and rational and orderly utilization of resources. The agricultural production not only meets the needs of modern people, but also meets the survival and development of future generations. The sustainable development trade system of agricultural trade is inseparably linked with society and the environment, and the integration of different dimensions into a systematic analysis is a current research hotspot. Such systematic research takes the production and trade of agricultural products as the carrier, including trade-resources-environment, trade-water-energy, trade-health, and so on.

According to Table 1, the CO_2_ complete emission coefficient of China's export trade can be obtained. In the horizontal sector comparison, the “electricity, gas, steam and air conditioning supply” had the highest CO_2_ complete emission coefficient and the largest change, which was from 34.01 kg/USD in 2019 to 15.79 kg/USD in 2021. The CO_2_ direct emission coefficient of “agriculture, forestry, animal husbandry and sideline fishery” was the lowest among all measured industries, but its change trend was different from other sectors. From 2018 to 2021, it showed a downward trend, which was from 1.81 kg/USD to 1.29 kg/USD. The direct CO_2_ emissions from export trade are shown in Table 1.

Agricultural production and agricultural environment have always been one of the research hotspots. Under the background of climate change, carbon emission has been recognized by experts and scholars as a proxy variable of agricultural production environmental pollution. The measurement of agricultural carbon emissions solves the problem that agricultural environmental pollution is difficult to quantify. In the past, agricultural environmental pollution was mostly studied by quantifying pesticides, chemical fertilizers, and unreasonable farming. Therefore, incorporating agricultural carbon emissions into the agricultural production performance evaluation framework enriches the existing theoretical basis of agricultural production and environmental protection. The research on the impact of trade on economic growth and the research on the impact of trade on the environment helps to clarify the mechanism of the impact of trade on agricultural economic growth and agricultural production environment. In addition, this paper measures agricultural carbon emission performance from the perspective of total factor productivity, so the research on the impact of trade on total factor productivity and green total factor productivity also has important reference significance for this paper.

In general, the trend of China's agricultural export trade is basically the same as the embodied carbon, showing an upward trend. From 2018 to 2019, the embodied carbon of China's agricultural export trade increased rapidly, from 7.14 mt to 15.62 mt, with an increase of 118.69%. In the same period, the trade volume increased from 4.609 billion yuan to 16.275 billion yuan, with an increase of 253.10%. The growth rate of implied carbon was smaller than that of trade volume. Among them, the growth rate of embodied carbon in exports was relatively obvious between 2017 and 2018 and from 2019 to 2020. From 2019 to 2020, the embodied carbon of China's agricultural export trade increased rapidly, from 6.23 mt to 8.94 mt, with an increase of 43.54%. In the same period, the trade volume increased from 4.293 billion yuan to 6.821 billion yuan, with an increase of 58.89%. From 2020 to 2021, the embodied carbon of China's agricultural export trade increased rapidly, from 11.39 mt to 15.82 mt, with an increase of 38.92%. In the same period, the trade volume rose from 9.736 billion yuan to 14.004 billion yuan, with an increase of 43.83%. The comparison of embodied carbon growth rate and trade volume is shown in Figure 5.

The direct cause of international trade between the two countries is the difference in product price caused by the difference in production costs between the two countries. That is, if there is still a price difference between the products of the two countries after deducting the export freight, the two countries can conduct international trade. The import trade of agricultural products is conducive to the introduction of clean technology. When agricultural trade develops to a certain extent, the competition of agricultural products will intensify, such as carbon emission taxes and fees, which will cause environmental costs to rise. Products with high agricultural carbon emission performance meet the needs of the market, and agricultural producers are forced to develop new technologies to accommodate low-carbon production requirements. The scale of agricultural trade expands the existing economies of scale, promotes technological progress, and guides changes in environmental regulations and policies, which may promote the use of carbon emission reduction technologies so as to reduce agricultural carbon emissions, improving agricultural carbon emissions performance. The expansion of the agricultural economic scale will increase the per capita income of agricultural producers, and people's requirements for the quality of the production environment will be further improved. Therefore, the willingness to purchase agricultural products with higher carbon emission performance begins to germinate, which promotes the progress and promotion of emission reduction technologies.

Overall, there are large differences in agricultural carbon emissions between provinces. Affected by the impact of imported products, the sales prices of agricultural products in various provinces and cities have decreased. Affected by this, agricultural exports expanded the most in province A ($19.62 million), province B ($20.44 million), province C ($21.33 million), province D ($32.86 million), and province E ($34.17 million). The five provinces with the largest changes in carbon emissions from agricultural exports are the same as the first three scenarios, namely, province G (81.95 million tons), province E (68.18 million tons), province F (66.44 million tons), province A (53.12 million tons), and province D (44.33 million tons). The United States imposed a 25% tariff on agricultural exports to China, while China lifted the tariffs on US agricultural products. The cumulative trade volume of agricultural exports and the carbon emissions of agricultural exports in various regions of China have increased, but the impact of the increase is very small. Compared with other provinces, the increase in carbon emissions from agricultural exports in provinces G and F increased significantly. The performance of agricultural carbon emissions and changes in agricultural products under the impact of imported agricultural products are shown in Table 2. Export trade is conducive to full interaction with consumers in the market, and new technologies and knowledge can be obtained in the process of interaction, which is conducive to the improvement and promotion of agricultural production technology.

As for imported products, if the trading partner countries have higher requirements for carbon emission standards, to a certain extent, it will give the exporting countries the motivation to promote the innovation and research and development of low-carbon technologies. For exporting countries, it is beneficial to reduce carbon dioxide emissions. From the perspective of countries, from 2022 to 2030, the Sino-US agricultural trade dispute will be detrimental to the economic growth of both countries. Under the scenario of mutual tariffs on agricultural products between the two countries, China's real GDP fell by 0.0218% cumulatively, which was higher than the 0.0015% decline in the United States over the same period. The Sino-US agricultural trade conflict is not conducive to the import and export trade of the two countries, but the decline in the United States is higher than that in China. After calculation, it is found that the scale of China's exports has decreased by 0.089%, which is lower than the decline of 0.361% in the United States. The trade conflict has a significant impact on China's import and export structure. Under the scenario of mutual tariffs on agricultural products, China's exports to the United States are expected to decrease by 6.28%, while China's imports from the United States will drop by 13.02% during the same period. Related to the negative economic impact, the Sino-US agricultural trade dispute will reduce the carbon emissions of the two countries by 0.013% and 0.024%, respectively.  Figure 6 shows the calculation of carbon emissions and agricultural economics in China and the United States. If the gap between economic interests can be broken, and intellectual property barriers can be eliminated, as well as the differences in technology and management levels between countries and regions can be reduced, then the technology transfer and the transformation of scientific and technological achievements between countries brought about by global cooperation will accelerate the elimination of carbon leakage in international trade. Therefore, it is necessary to formulate a reasonable agricultural carbon emission performance evaluation system to provide policy guidance and institutional guarantee for evaluating the coordinated development of China's agricultural production and agricultural environment. At present, most of China's low-carbon production work focuses on industrial emission reduction. Although industrial carbon reduction has achieved results, insufficient attention has been paid to agricultural carbon emissions, and agricultural production models with high energy consumption, high investment, and low efficiency still exist. Agricultural production in some areas is still in a nonrecyclable state.

## 9. Conclusion

With the consolidation of China's international status, China's import and export trade has made great progress compared with investment and consumption. For agricultural production, the level of agricultural carbon emission performance is an important indicator to measure whether agricultural production is of high quality and meets green standards. The high-carbon production of agricultural products faces the threat of carbon tariffs in developed countries, so reduces agricultural carbon emissions and increases the import of agricultural products on the premise of ensuring food security. The high-carbon production of agricultural products faces the threat of carbon tariffs in developed countries, so agricultural carbon emissions are reduced. Under the premise of ensuring food security, the import of agricultural products has been increased. This paper takes agricultural trade as the research object, analyzes the resource flow and carbon emissions behind the trade, and combines the trade, resources, and environmental systems for analysis to provide a research basis for sustainable development. This paper makes an objective evaluation and analysis of China's agricultural development of carbon finance from the actual point of view, which provides a more feasible theoretical basis and policy ideas for the development of carbon finance in the field of the agricultural economy. Under the background of global climate and environmental change, the research on agricultural production development policy oriented toward low-carbon and high-efficiency is not only a hot spot concerned by all countries in the world, but also an important strategic issue related to the development of China's low-carbon agricultural economy. However, this study does not further analyze the factors of carbon dioxide emissions. The work in the future can further explore the development of carbon finance in the field of the agricultural economy.

## Figures and Tables

**Figure 1:** Impact of agricultural trade liberalization on the agricultural environment.

**Figure 2:** Theoretical analysis model of the relationship between agricultural carbon emissions and agricultural economic growth.

**Figure 3:** China's agricultural products export survey. (a) Vegetables, aquatic products, fruits, livestock products, and beverages. (b) Grain products, oilseeds, sugar, nuts, and other agricultural products.

**Figure 4:** China's agricultural product import surveys. (a) Aquatic products, vegetable oils, beverages, grains, and fruits. (b) Cotton and linen silk, grain products, other products, oilseeds, and animal products.

**Figure 5:** Comparison of embodied carbon growth rate and trade volume.

**Figure 6:** China and the United States carbon emissions and agricultural economic calculation.

**Table 1:** Direct CO_2_ emissions from export trade.

Department	2018	2019	2020	2021
Agriculture, forestry, animal husbandry, and fishery (kg/dollar)	0.38	0.33	0.35	0.31
Mining industry (kg/dollar)	1.70	1.11	0.89	0.81
Food, beverage, and tobacco products (kg/dollar)	0.69	0.31	0.13	0.11
Textile industry (kg/dollar)	0.51	0.18	0.13	0.16

**Table 2:** Agricultural carbon emission performance and changes in agricultural products under the impact of imported agricultural products.

Different provinces	Changes in cumulative agricultural exports (USD million)	Carbon emissions (million tons)
A	19.62	53.12
B	20.44	15.22
C	21.33	10.33
D	32.86	44.33
E	34.17	68.18
F	12.15	66.44
G	14.32	81.95

## Data Availability

The data used to support the findings of this study are available from the corresponding author upon request.
